The article "Efficacy of CAD/CAM Technology in Interventions Implemented in Orthodontics: A Scoping Review of Clinical Trials" was published in 2022. Journal: Biomed Res Int.

# Efficacy of CAD/CAM Technology in Interventions Implemented in Orthodontics: A Scoping Review of Clinical Trials

**DOI:** 10.1155/2022/5310555

**Published:** 2022-06-02

**Authors:** Carlos M. Ardila, Andrés Elorza-Durán, Daniel Arrubla-Escobar

**Affiliations:** ^1^Biomedical Stomatology Research Group, Universidad de Antioquia, U de A, Medellín, Colombia; ^2^Institución Universitaria Visión de Las Américas, Medellín, Colombia

## Abstract

**Objectives:**

To evaluate the efficacy of computer-aided design/computer-aided manufacturing (CAD/CAM) technology in interventions implemented in orthodontics.

**Methods:**

A scoping review of scientific evidence was accomplished, involving different databases. MesH terms and keywords were provided to examine clinical trials (CTs) in all languages. Exclusively CTs that fulfilled the eligibility criteria were admitted.

**Results:**

Eight CTs were chosen. These experiments evaluated 542 patients. Four CTs compared the computer-aided indirect bonding method versus the traditional direct bonding of orthodontic brackets. Three CTs compared CAD/CAM retainers with other types of retainers, and one CT compared the CAD/CAM group with multistranded stainless steel wires versus stainless steel wires. Regarding the efficacy of the interventions with CAD/CAM technology used in orthodontics, variable results were found. The indirect bonded customized CAD/CAM brackets presented just a slight effect on the treatment efficacy and therapy results. Two CTs showed that an indirect bonding self-ligating standard system had a similar quality of therapy in comparison with the CAD/CAM customized bracket system. Concerning the clinical failure rate, no differences were presented between the CAD/CAM retainer and other retainers. A CAD/CAM system had more loose brackets than a noncustomized system and was observed also a greater amount of immediate debonding with CAD/CAM indirect bonding than with direct bonding. CAD/CAM fixed retainers revealed inferior relapse and fewer failures than lab-based and conventional chairside retainers. No changes between treatment groups were observed regarding the total therapy time, amount of appointments, and quantity of archwire bends.

**Conclusions:**

In general terms, no greater efficacy of CAD/CAM technology was observed over traditional therapies used in orthodontics. However, it was found that gingival inflammation and the accumulation of bacterial plaque and dental calculus were lower when CAD/CAM retainers were used. When comparing interventions that include CAD/CAM systems with conventional therapies, no significant reduction in care times was found.

## 1. Introduction

The advent of computer-aided design/computer-aided manufacturing (CAD/CAM) technology has brought much innovation to dentistry. In orthodontics, this technology has been incorporated during diagnosis and treatment plans. CAD/CAM technology facilitates a fully digital workflow; moreover, various protocol studies have postulated clinical reliability, and it has been indicated that this technology produces very favorable feedback from patients [1, 2]. A retrospective study also proposed that CAD/CAM applications reduced treatment time [3].

The article "Efficacy of CAD/CAM Technology in Interventions Implemented in Orthodontics: A Scoping Review of Clinical Trials" was published in 2022. Journal: Biomed Res Int.

Regarding fixed purposes, CAD/CAM technology may promote the accuracy of bracket placement, considering that its location significantly influences treatment effects [4]. Some fully individualized bracket systems incorporate virtual configurations to assume treatment outcomes, taking into account individual tooth surface and morphology, and custom archwires [5]. Furthermore, patients treated with CAD/CAM orthodontic systems, in a retrospective study, required fewer appointments for archwire changes; besides, the treatment time was shorter and presented an inferior American Board of Orthodontics (ABO) score [6].

The CAD/CAM technology has also made it possible to develop retainers. The CAD/CAM lingual retainer is placed digitally, giving a particularly improved position, greater precision of fit, and interproximal adaptation. It causes less irritability of the tongue and prevents occlusal interferences. The rectangular nickel-titanium archwire offers better flexibility, improving the physiological movement of the teeth. Moreover, the wire is electropolished, making it smooth and corrosive resistant, reducing the growth of bacterial plaque [7].

Computer technology has also permitted novel methods of indirect bonding. The brackets are positioned in a virtual 3D dental model; then, this technology generates information on its location, and subsequently, this is indirectly transferred to the teeth. A prototype procedure indicated the reduction of the time of dental consultation and the improvement of precision [8].

Assessing the best available scientific evidence through clinical trials that compare CAD/CAM technologies with conventional therapies will allow clinicians to make better decisions in their practice. In this context, it is relevant to carry out a scoping review of clinical trials, which allows for evaluating the efficacy of CAD/CAM technology in interventions implemented in orthodontics. To achieve this objective, it was proposed to answer some questions related to the efficacy, treatment times, benefits, and/or adverse events of therapies using CAD/CAM in orthodontics.

## 2. Materials and Methods

This review of clinical trials was carried out considering the PRISMA (Preferred Reporting Items for Systematic Reviews and Meta-analyses) extension for scoping reviews [9]. The scoping structure involved different databases such as SCOPUS, PubMed/MEDLINE, SCIELO, and LILACS, including the gray literature. MesH terms and keywords were provided to examine clinical trials in humans in all languages, with no publication date range, including the terms computer-aided design, CAD/CAM system, 3D treatment planning, orthodontic, orthodontic treatment, customized brackets, retainer, digital orthodontics, intervention studies, and clinical trial. Trials comparing interventions between CAD/CAM groups were discarded. Exclusively clinical trials (CTs) that fulfilled the eligibility criteria were admitted. Research related to case reports, case series, duplicate studies, in vitro experiments, and animal studies were excluded.

The article "Efficacy of CAD/CAM Technology in Interventions Implemented in Orthodontics: A Scoping Review of Clinical Trials" was published in 2022. Journal: Biomed Res Int.

### 2.1. Questions

This scoping review aims to answer the following questions: In which areas of orthodontics are CAD/CAM systems used for interventions? Do interventions with CAD/CAM technology show greater efficacy? Do interventions with CAD/CAM technology require less time? Do CAD/CAM interventions present benefits or adverse events?

### 2.2. Review Process

Two investigators reviewed the titles and abstracts and selected CTs to assess the full text for potential eligibility. In case of disagreement between authors, trial eligibility was made by consensus. The Kappa statistical test was used to assess the value of agreement between observers (>95).

### 2.3. Data Collection

A table was designed to incorporate the most relevant data from the selected CTs. This process was performed independently by each of the researchers. Subsequently, the data were compared. Recorded data included authors' names, date of publication, age and gender of participants, number of participants, intervention, and control, comparison between the groups (main studied variables), and treatment time.

### 2.4. Risk of Bias

The risk of bias and quality assessment of the included trials was performed following the Jadad scale for CTs [10], by two authors.

## 3. Results

The electronic search yielded 46 studies. After reviewing the titles and abstracts, 33 investigations were excluded. Reading the full text resulted in the exclusion of 5 additional trials. Finally, 8 CTs [5, 11–17] were included in this scoping review (Figure 1).

The characteristics of the included studies are presented in Table 1. Three CTs were randomized single-blind, controlled, and with parallel design [11, 12, 17]. Three CTs were randomized unblinded, controlled, and with parallel design [14–16], one CT was randomized unblinded, controlled, and with split-mouth design [13], and one CT was quasi-randomized, controlled, with parallel design [5]. One CT compared 4 groups [14], 2 CTs compared 3 groups [11, 12], and 5 CTs compared 2 groups [5, 13, 15–17]. These CTs were published between 2017 and 2022.

The article "Efficacy of CAD/CAM Technology in Interventions Implemented in Orthodontics: A Scoping Review of Clinical Trials" was published in 2022. Journal: Biomed Res Int.

These trials assessed 542 patients with a minimum sample of 24 patients [15] and a maximum of 174 [16]. These experiments evaluated different interventions in orthodontics. Four studies compared the computer-aided indirect bonding method versus the traditional direct bonding of orthodontic brackets [5, 13, 15, 16]. Three studies compared CAD/CAM retainers with other types of retainers [12, 14, 17], and one CT compared CAD/CAM group with multistranded stainless steel wires versus stainless steel Ortho-FlexTech wires group (traditional group) and Lab group with multistranded stainless steel wires [11].

Variable results were found regarding the efficacy of interventions with CAD/CAM technology used in orthodontics. In contrast with a direct bonded self-ligating bracket system, the utilization of indirect bonded customized CAD/CAM brackets presented just a slight effect on treatment efficacy. Besides, after therapy, the ABO score in both interventions was diminished, without significant differences [5]. Likewise, an indirect bonding self-ligating standard system showed a similar quality of therapy in comparison with the CAD/CAM customized bracket system, and the final ABO score was similar [15]. Penning et al. [16] also showed that the treatment quality was equivalent between customized orthodontic systems and noncustomized orthodontic systems. Concerning the clinical failure rate, no differences were presented between the CAD/CAM retainer and other retainers, admitting that CAD/CAM retainer has better fitting precision [12, 17]. Furthermore, the Little's irregularity index for CAD/CAM group was less than that of the other groups but similar to the stainless steel retainers [14, 17]. In contrast, a customized orthodontic system had more loose brackets than a noncustomized system [16] and was observed also a greater amount of immediate debonding with CAD/CAM indirect bonding than with direct bonding [13]. Regarding bonding fixed retainers, CAD/CAM fixed retainers revealed inferior relapse than lab-based and conventional chairside retainers. The CAD/CAM retainers also showed fewer failures than lab-based retainers [11].

Considering the time spent during the interventions, the results were also variable. It was founded that while CAD/CAM indirect bonding proved less chair time, the total bonding period, counting digital bracket position, was larger than for direct bonding [13]. It was also observed that the indirect bonding self-ligating standard system had a 26% longer total orthodontic therapy period, in comparison with the CAD/CAM customized bracket system [15]. Instead, Hegele et al. [5], Adanur et al. [14], and Penning et al. [16] did not find differences in treatment time between the analyzed groups.

The article "Efficacy of CAD/CAM Technology in Interventions Implemented in Orthodontics: A Scoping Review of Clinical Trials" was published in 2022. Journal: Biomed Res Int.

Responding to the fourth question of this scoping review, it was found that gingival inflammation and the accumulation of bacterial plaque and dental calculus were lower when CAD/CAM retainers were used [12, 14]; however, Alrawas et al. [12] and Gelin et al. [17] did not show statistically significant differences between groups. On the other hand, two CTs revised here indicated that CAD/CAM indirect bonding was more expensive than direct bonding [13, 16]. Penning et al. [16] denoted that the patients in the customized group had more complaints. The rest of the clinical trials evaluated in this scoping review did not report adverse events with the use of CAD/CAM technology.

Two studies had a high risk of bias [5, 15], while the rest of the selected trials had a moderate risk of bias (Table 2).

## 4. Discussion

To the best of the authors' understanding, this scoping review is the first to compare the efficacy of CAD/CAM technology used in orthodontics with conventional therapies. Considering that the new CAD/CAM technologies propose novelties related to clinical interventions performed in orthodontics, it is essential to evaluate their clinical efficacy with the best available scientific evidence. Taking this aspect into account, in this review, answers were given to each of the four proposed questions.

In contrast with a direct bonded self-ligating bracket system, the utilization of indirect bonded customized CAD/CAM brackets presented just a slight effect on treatment efficacy and therapy results. Besides, after therapy, two trials revised here showed that the ABO score in both interventions was diminished, without significant differences [5, 15]. These findings corroborated previous results of a retrospective study that presented no changes between indirectly bonded CAD/CAM brackets, indirectly bonded custom brackets, and directly bonded custom brackets [3].

In this review, the study by Czolgoz et al. [13] showed that CAD/CAM indirect bonding presented more immediate bonding failures than conventional direct bonding. Comparable results were also documented by Penning et al. [16]. It has been postulated that indirect bonding failures may be caused by short periods of light-curing time [13].

Two CTS in this review showed that a customized orthodontic system had more loose brackets than a non-customized system [16] and it was observed also a greater amount of immediate debonding with CAD/CAM indirect bonding than with direct bonding [13]. Even though it is expected that a customized bracket has an ideal fit, the customized and the noncustomized system differ in the personally computed location of the bracket slot; then, the design of the personalized bracket is bigger, facilitating debonding [16]. Moreover, the customized brackets were indirectly bonded, characteristics that have also caused higher failure rates in a previous study [18].

The article "Efficacy of CAD/CAM Technology in Interventions Implemented in Orthodontics: A Scoping Review of Clinical Trials" was published in 2022. Journal: Biomed Res Int.

The trial by Alrawas et al. [12] showed no differences between the CAD/CAM retainer and other retainers, which corresponds with the report of Geling et al. [17] and Attack et al. [19] and diverges with the research of Al-Moghrabi et al. [20], who established that the fixed retainers have higher efficacy, considering that patients are less collaborative over time with the use of removable retainers.

Regarding bonding fixed retainers, CAD/CAM fixed retainers revealed inferior relapse than lab-based and conventional chairside retainers. The CAD/CAM retainers also showed fewer failures than lab-based retainers. The CAD/CAM and lab groups utilized more rigid dentaflex wires; moreover, they are subject to constant deformation in comparison with Ortho-FlexTech wires that are flexible [11]. Similarly, thicker and rigid wires have been reported to better maintain intercanine width than flexible wires [21].

This review found that CAD/CAM indirect bonding (clinical chair time plus digital bracket location time) was larger than direct bonding [13]. A comparative study also presented a greater total indirect bonding time [22]. However, retrospective studies with small simple sizes revealed a diminution in therapy time and quantity of appointments for the CAD/CAM systems [3, 6]. Similarly, Xiaolei et al. [23] indicated that the digital method was more effective in lingual retainer construction than the standard process. Moreover, it was more difficult to fabricate a lingual retainer for the maxilla than for the mandible; the standard technique cost two times to bend the lingual retainer for the maxilla of the time to bend the lingual retainer for the mandible. Instead, in this review, Hegele et al. [5], Adanur et al. [14], and Penning et al. [16] did not find differences in treatment time between the analyzed groups. These controversial results may have several explanations. Implementing a novel technique during clinical care is not constantly simple. The clinician's expertise with a new software increases with the passing of the practice, an aspect that can impact the results [13, 16]. On the other hand, the epidemiological design, the objectives, the interventions compared, the definition of chronological order, and the selection criteria of the studies may cause differences in the results [5].

The article "Efficacy of CAD/CAM Technology in Interventions Implemented in Orthodontics: A Scoping Review of Clinical Trials" was published in 2022. Journal: Biomed Res Int.

Traditionally, it has been indicated that the indicators of bacterial plaque accumulation and gingival inflammation are higher with the use of stainless steel retainers [24]. The smoothness and polish of CAD/CAM retainers allow less plaque accumulation and therefore less inflammation, aspects that were corroborated in this review [12, 14].

A clinical trial selected in this review indicated that the costs of CAD/CAM technology are slightly higher than those of an orthodontist using conventional treatments [13]. Penning et al. [16] indicated that this is because CAD/CAM technology is more expensive due to laboratory costs. However, the costs of CAD/CAM technology present controversial results in other specialties of dentistry. Some studies indicate that the costs are similar to conventional treatments, while others indicate that the values are lower [25, 26]. More cost-effectiveness studies are required when using CAD/CAM systems in orthodontics to present more conclusive results in this regard.

In this scoping review, only one trial reported patient complaints related to the thickness of customized brackets [16]. Other studies have also described patient complaints in other areas of dentistry when this technology has been implemented [27, 28].

The main limitation of this scoping review is related to the moderate and high risk of bias of the CTs selected. Most of the biases in these studies were related to double-blinding. It has been reported that blinding the patient and the clinician in orthodontic interventions is difficult [5]. However, a greater number of CTs with a low risk of bias are required to allow more conclusive results. Other limitations of this review are related to missing keywords and other databases. However, two of the most important databases were used.

Finally, it is necessary to design clinical trials with longer follow-up times, higher scientific quality, and low risks of bias, to obtain more reliable results about CAD/CAM technologies used in orthodontics. Furthermore, the cost-benefit and patient satisfaction with the use of these technologies should also be investigated.

## 5. Conclusions

In general terms, no greater efficacy of CAD/CAM technology was observed over traditional therapies used in orthodontics. However, it was found that gingival inflammation and the accumulation of bacterial plaque and dental calculus were lower when CAD/CAM retainers were used. When comparing interventions that include CAD/CAM systems with conventional therapies, no significant reduction in care times was found.

The article "Efficacy of CAD/CAM Technology in Interventions Implemented in Orthodontics: A Scoping Review of Clinical Trials" was published in 2022. Journal: Biomed Res Int.

## Figures and Tables

**Figure 1:** Flowchart of the CTs selection method.

**Table 1:** Features of the CTs evaluated.

Authors Publication date	Participants	Mean Age	Female Male	Intervention control	Main outcomes	Treatment time
Shim et al. 2022	46	16 years	28/18	CAD/CAM group with multistranded stainless steel wires versus lab group with multistranded stainless steel wires versus a group with stainless steel Ortho-FlexTech wires (traditional group)	The CAD/CAM group experienced a less intercanine width decrease (*P* < 0.05). The CAD/CAM group experienced a less increase in Little's irregularity index (*P* < 0.05). Failures from greatest to least were experienced by the lab group (43.8%), the CAD/CAM group (25%), and the traditional group (14.3%)	6 months of bonding fixed retainers
Adanur-Atmaca et al. 2021	132	16 years	92/40	Lingual retainers with 0.016 3 0.022 in dead soft wire versus Lingual retainers with 0.0215 in 5 strand stainless steel wire versus lingual retainers with 0.014 3 0.014-in CAD/CAM nitinol versus lingual retainers with connected bonding pads	Gingival inflammation and calculus accumulation were the lowest in CAD/CAM group (*P* < 0.05). The Little's irregularity for CAD/CAM group and stainless steel retainers was less than that of the other groups. No clinically significant worsening of periodontal health or relapse was seen in any groups after 1 year	12 months
Hegele et al. 2021	38	14 years	23/15	Indirect bonded customized CAD/CAM brackets versus direct bonded self-ligating brackets	No differences between both treatment groups were found concerning overall treatment time, the number of appointments, and the number of archwire bends. Bonding failures occurred more often using the CAD/CAM system. Indirectly bonded brackets did not have to be repositioned as often as directly bonded brackets. Treatment results with both systems were similar concerning their effects on the reduction of ABO score. The number of the used archwires was higher in the CAD/CAM group	16.7 months
Jackers et al. 2021	24	23 years	17/7	CAD/CAM custom indirect bonding self-ligating system versus indirect bonding self-ligating standard system	The indirect bonding self-ligating standard system had a 26% longer overall orthodontic treatment time compared with the CAD/CAM customized bracket system (*P* = 0.00002). The indirect bonding self-ligating bracket system demonstrated the same quality of treatment. Patients showed a high level of acceptance and satisfaction with both techniques	393 days in the CAD/CAM group 497 days in the standard system
Alrawas et al. 2021	60	20 years	43/17	CAD/CAM NiTi retainer, multistranded stainless steel versus single-stranded nickel-free titanium retainer versus vacuum-formed removable group	All groups showed some relapse in the lower anterior teeth. No statistical significance was found intergroup in terms of all measured values. Less plaque accumulation and gingival inflammation were observed in the CAD/CAM NiTi retainer group but without statistical significance	6 months of follow-up
Czolgosz et al. 2020	27	17 years	15/12	Computer-aided indirect bonding method versus traditional direct bonding of orthodontic brackets	Clinical chair time for bonding half a mouth was significantly shorter for computer-aided indirect bonding (*P* < 0.001). There was no single immediate debonding with the direct bonding method, while 14 brackets were lost with the indirect bonding method (*P* = 0.0001). Cost-minimization analysis showed that computer-aided indirect bonding was more expensive than direct bonding	Not reported
Gelin et al. 2020	41	17 years	43/18	To compare CAD/CAM customized nitinol retainers with standard stainless-steel fixed retainers	No significant difference between customized CAD/CAM nickel-titanium lingual retainers and standard stainless-steel lingual retainers in terms of dental anterior stability and retainer survival were observed. Both retainers eventually appeared to be equally effective in maintaining periodontal health	12 months
Penning et al. 2017	174	14 years	103/71	Customized orthodontic system versus non-customized orthodontic system	The customized group had more loose brackets, a longer planning time, and more complaints (*P* < 0.05). The customized orthodontic system was not associated with significantly reduced treatment duration, and treatment quality was comparable between the 2 systems	1.29 years in the customized system 1.24 years in the non-customized system

The article "Efficacy of CAD/CAM Technology in Interventions Implemented in Orthodontics: A Scoping Review of Clinical Trials" was published in 2022. Journal: Biomed Res Int.

**Table 2:** Quality of the selected studies (Jadad et al. 1996).

Clinical trial	Randomization	Double blinding	Withdraw	Proper randomization	Proper double blinding	Score
Shim et al. (2022)	1	0	1	1	0	3
Adanur-Atmaca et al. (2021)	1	0	1	1	0	3
Hegele et al. (2021)	0	0	0	0	0	0
Jackers et al. (2021^)^	1	0	1	0	0	2
Alrawas et al. (2021)	1	0	1	1	0	3
Czolgosz et al. (2020^)^	1	0	1	1	0	3
Gelin et al. (2020)	1	0	1	1	0	3
Penning et al. (2017)	1	0	1	1	0	3

## Data Availability

Records were obtained from the included investigations.
